The article "Large tumor suppressor kinase 2 overexpression attenuates 5-FU-resistance in colorectal cancer via activating the JNK-MIEF1-mitochondrial division pathway" was retracted in 2023. Reasons: duplicated images; signs of a paper mill; unreliable data; unreliable results or conclusions.

# Large tumor suppressor kinase 2 overexpression attenuates 5-FU-resistance in colorectal cancer via activating the JNK-MIEF1-mitochondrial division pathway

**DOI:** 10.1186/s12935-019-0812-3

**Published:** 2019-04-11

**Authors:** Weilong Yao, Shengtao Zhu, Peng Li, Shutian Zhang

**Affiliations:** Department of Gastroenterology, Beijing Friendship Hospital, Capital Medical University, National Clinical Research Center for Digestive Disease, Beijing Digestive Disease Center, Beijing Key Laboratory for Precancerous Lesion of Digestive Disease, No. 95, Yong’an Road, Xicheng District, Beijing, 100050 People’s Republic of China

**Keywords:** 5-FU, Colorectal cancer, LATS2, Mitochondrial fission, MIEF1, Apoptosis

## Abstract

**Background:**

5-Fluorouracil (5-FU) is a standard treatment for colorectal cancer, but most patients develop 5-FU resistance. Here, we conducted experiments to identify an effective approach to augment 5-FU-based treatment in colorectal cancer in vitro.

**Methods:**

SW480 cells were in the present study and treated with 5-FU. Besides, LATS2 adenovirus vectors were infected into SW480 cells. Western blotting, immunofluorescence and ELISA were used to evaluate cell death and mitochondrial function. Pathway blocker was used to verify the role of MAPK-JNK pathway in SW480 cell death.

**Results:**

An obvious drop in large tumor suppressor kinase 2 (LATS2) expression was observed in SW480 cells after treatment with 5-FU. In addition, upregulation of LATS2 expression through infection with LATS2 adenovirus further increased the reduction of SW480 cell viability induced by 5-FU. Functional exploration showed that 5-FU treatment suppressed mitochondrial membrane potential, enhanced cyt-c release into the nucleus, induced an oxidative injury environment by promoting ROS production, and eventually upregulated Bax-related mitochondrial apoptosis. Besides, LATS2 overexpression in combination with 5-FU treatment further perturbed mitochondrial homeostasis, and this effect was achieved by elevating mitochondrial division. Mechanistically, LATS2 overexpression and 5-FU co-treatment amplified mitochondrial division by upregulating MIEF1 expression in a manner dependent on MAPK-JNK axis. Knockdown of MIEF1 using an siRNA-mediated loss of function assay and/or inhibition of the MAPK-JNK pathway using the specific inhibitor SP600125 abolished LATS2/5-FU-mediated deleterious effects on mitochondrial performance and SW480 cell viability.

**Conclusions:**

In light of the above findings, LATS2 downregulation could be a potential mechanism of low response to 5-FU treatment. Overexpression of LATS2 to further disrupt mitochondrial function via the JNK-MIEF1 signalling pathway might be a method to optimize 5-FU-based chemotherapy.

The article "Large tumor suppressor kinase 2 overexpression attenuates 5-FU-resistance in colorectal cancer via activating the JNK-MIEF1-mitochondrial division pathway" was retracted in 2023. Reasons: duplicated images; signs of a paper mill; unreliable data; unreliable results or conclusions.

## Background

Colorectal cancer (CRC) is the third leading cause of cancer-related deaths worldwide due to its poor prognosis [1]. Although several advancements have been made in the diagnosis and treatment (radiation therapy and chemotherapy) of CRC, the 5-year survival rate is only ~ 60% [2, 3]. Currently, the first-line anti-cancer approach for patients with CRC is surgery in combination with chemotherapeutic regimens such as 5-fluorouracil (5-FU) or leucovorin. However, due to the acquisition of resistance, the cancer-killing effect of 5-FU is inevitably attenuated, as evidenced by increased CRC cell survival and rapid metastasis. Accordingly, there is an urgent need to identify the core mechanisms responsible for acquired 5-FU resistance in CRC to augment clinical benefits in patients with CRC.

Mitochondrial division plays a key role in controlling cancer fate. Oxidative stress due to the accumulation of ROS, which primarily originate from excessive mitochondrial division, impairs cancer viability and promotes cell senescence [4, 5]. In addition, massive mitochondrial division has been found to amplify death execution through the release of pro-apoptotic proteins (such as cyt-c) in the nucleus [6, 7]. Numerous studies have reported that mitochondrial division could be considered an effective means of further augmenting the therapeutic sensitivity of CRC [8]. However, the upstream mediator of mitochondrial division in CRC remains unknown. Recently, mitochondrial elongation factor 1 (MIEF1) was identified as a potential novel mitochondrial division mediator [9]. Higher expression of MIEF1 has been observed in models of brain ischemia reperfusion injury [10] and ultraviolet irradiation-induced epidermal injury [9]. However, the biological role of MIEF1-related mitochondrial division in 5-FU resistance is not fully understood.

The large tumor suppressor kinase 2 (LATS2)-Hippo pathway is attracting research interest, as several cancer biological functions are closely modulated by the LATS2-Hippo pathway, such as cancer cycle regulation, differentiation, movement, survival and metastasis [11]. In osteosarcoma, LATS2 levels are considered a prognostic factor for cancer recurrence [11]. In lung cancer, LATS2 overexpression activates mitochondrial fission, which promotes cancer death [12]. In liver cancer, LATS2 controls the epithelial-mesenchymal transition in an miR-650-dependent manner [13]. The cancer metabolic state and tumour differentiation [14] are also regulated by LATS2. However, few studies have explored the influence of LATS2 in 5-FU-treated CRC. In the present study, we explore whether LATS2 is involved in therapeutic resistance via modulating MIEF1-related mitochondrial division in 5-FU-treated CRC.

The article "Large tumor suppressor kinase 2 overexpression attenuates 5-FU-resistance in colorectal cancer via activating the JNK-MIEF1-mitochondrial division pathway" was retracted in 2023. Reasons: duplicated images; signs of a paper mill; unreliable data; unreliable results or conclusions.

## Methods and material

### Cell culture and transfection

SW480 colorectal cancer cells (ATCC^®^ CCL-228™) were purchased from the National Infrastructure of Cell Line Resource (Beijing, China). All these cells were grown in RPMI-1640 medium supplemented with 10% foetal bovine serum (FBS, Gibco, Grand Island, NY, USA) at 37 °C in a humidified atmosphere of 95% air and 5% CO_2_. SW480 cells were treated with different doses of 5-FU for 12 h according to a previous study [15]. The siRNA against MIEF1 and the pDC315-LATS2 vector were obtained from GenePharm (Shanghai, China). Meanwhile, transfection was performed using Lipofectamine 2000 (Invitrogen; Thermo Fisher Scientific, Inc.) following the manufacturer’s instructions [16]. After 6 h, the cells were transferred to complete growth medium, and 48 h later, the cells were harvested and used for further experiments. The siRNA knockdown efficiency and overexpression efficiency were confirmed via western blotting [17].

### Western blotting

Total protein was extracted by RIPA (R0010, Solarbio Science and Technology, Beijing, China), and the protein concentration of each sample was detected with a bicinchoninic acid (BCA) kit (20201ES76, Yeasen Biotech Co., Ltd, Shanghai, China) [18]. Deionized water was added to generate 30-µg protein samples for each lane. A 10% sodium dodecyl sulphate (SDS) separation gel and concentration gel were prepared [19]. The following diluted primary antibodies were added to the membrane and incubated overnight: Bcl2 (1:1000, Cell Signaling Technology, #3498), Bax (1:1000, Cell Signaling Technology, #2772), caspase-9 (1:1000, Cell Signaling Technology, #9504), survivin (1:1000, Cell Signaling Technology, #2808), Cyclin D (1:1000, Abcam, #ab134175), CDK4 (1:1000, Abcam, #ab137675), complex III subunit core (CIII-core2, 1:1000, Invitrogen, #459220), complex II (CII-30, 1:1000, Abcam, #ab110410), complex IV subunit II (CIV-II, 1:1000, Abcam, #ab110268), Drp1 (1:1000, Abcam, #ab56788), Fis1 (1:1000, Abcam, #ab71498), Opa1 (1:1000, Abcam, #ab42364), Mfn2 (1:1000, Abcam, #ab56889), Mff (1:1000, Cell Signaling Technology, #86668), LATS2 (1:1000, Abcam, #ab135794), MIEF1 (1:1000, Abcam, #ab89944), JNK (1:1000; Cell Signaling Technology, #4672), p-JNK (1:1000; Cell Signaling Technology, #9251) [20].

### Quantitative PCR

TRIzol reagent (Invitrogen; Thermo Fisher Scientific, Inc.) was used to isolate total RNA from cells. Subsequently, the Reverse Transcription kit (Kaneka Eurogentec S.A., Seraing, Belgium) was applied to transcribe RNA (1 μg in each group) into cDNA at room temperature (~ 25 °C) for 30 min [21]. The qPCR was performed with primers using SYBR™ Green PCR Master Mix (Thermo Fisher Scientific, Inc. Cat. No. 4309155) [22].

The article "Large tumor suppressor kinase 2 overexpression attenuates 5-FU-resistance in colorectal cancer via activating the JNK-MIEF1-mitochondrial division pathway" was retracted in 2023. Reasons: duplicated images; signs of a paper mill; unreliable data; unreliable results or conclusions.

### ELISA

The Caspase 9 Activity Assay Kit (Beyotime, China, Cat. No: C1158) was used to measure the activity of caspase-9 according to the manufacturer’s instructions [23]. The concentrations of GSH, SOD and GPX were evaluated using commercial kits (Cellular Glutathione Peroxidase Assay Kit, Beyotime, China, Cat. No: S0056; Glutathione Reductase Assay Kit, Beyotime, China, Cat. No: S0055; Total Superoxide Dismutase Assay Kit, Beyotime, China, Cat. No: S0101, respectively) [24]. ATP production was measured using a luciferase-based ATP assay kit (Beyotime Institute of Biotechnology) with a microplate reader [25].

### Cell proliferation assay and MTT assay

Cellular proliferation was evaluated via EdU assay. Cells were seeded onto a 6-well plate, and the Cell-Light™ EdU Apollo^®^567 In Vitro Imaging Kit (Thermo Fisher Scientific Inc., Waltham, MA, USA; Catalogue No. A10044) was used to observe the EdU-positive cells according to the manufacturer’s instructions [26]. MTT assay was used to observe the cellular viability. Cells were seeded onto a 96-well plate, and the MTT was then added to the medium (2 mg/ml; Sigma-Aldrich) [27]. Subsequently, the cells were cultured in the dark for 4 h, and DMSO was added to the medium. The OD of each well was observed at A490 nm via a spectrophotometer (Epoch 2; BioTek Instruments, Inc., Winooski, VT, USA) [28].

### Terminal deoxynucleotidyl transferase-mediated deoxyuridine triphosphate-biotin nick end labelling (TUNEL) staining

To perform the TUNEL assay, cells were fixed in 4% paraformaldehyde at room temperature for 30 min [29]. After that, a TUNEL kit (Roche Apoptosis Detection Kit, Roche, Mannheim, Germany) was used on the slices according to the instructions [30]. Finally, the sections were amplified to 400×; the apoptotic cells in at least 10 fields were randomly chosen. The apoptotic index was the proportion of apoptotic cells to total cells according to a previous study [31].

### Transwell assay

Transwell units were used to evaluate the migratory response of cells. A total of 1 × 10^3^ cells were added to the upper chamber inside the transwell units [32]. Then, RPMI-1640 supplemented with 10% foetal bovine serum was added to the lower chamber inside the transwell unites. After 12 h, the upper chamber was isolated, and the migrated cells were fixed with 4% paraformaldehyde at room temperature for 30 min [33]. Subsequently, migrated cells were treated with 0.1% crystal violet at room temperature for 30 min. Finally, the migrated cells in at least 10 fields were randomly chosen and recorded with a digital microscope system (IX81, Olympus) [34].

The article "Large tumor suppressor kinase 2 overexpression attenuates 5-FU-resistance in colorectal cancer via activating the JNK-MIEF1-mitochondrial division pathway" was retracted in 2023. Reasons: duplicated images; signs of a paper mill; unreliable data; unreliable results or conclusions.

### Fluorescence microscopy

Cells were plated on glass slides in a 6-well plate at a density of 1 × 10^6^ cells per well. Subsequently, cells were fixed in ice-cold 4% paraformaldehyde for 30 min, permeabilized with 0.1% Triton X-100, and blocked with 2% gelatine in PBS at room temperature [35]. The cells were then incubated with the primary antibodies: Tom20 (1:1000, Abcam, #ab186735), MIEF1 (1:1000, Abcam, #ab89944), p-JNK (1:1000; Cell Signaling Technology, #9251) and cyt-c (1:500; Abcam; #ab90529) [36].

### Mitochondrial membrane potential measurement and ATP detection

Mitochondrial membrane potential was measured with JC-1 assays (Thermo Fisher Scientific Inc., Waltham, MA, USA; Catalogue No. M34152). Cells were treated with 5 mM JC-1 and then cultured in the dark for 30 min at 37 °C [37]. Subsequently, cold PBS was used to remove the free JC-1, and DAPI was used to stain the nucleus in the dark for 3 min at 37 °C. The mitochondrial membrane potential was observed under a digital microscope (IX81, Olympus) [38]. Cellular ATP content was measured according to a previous report via ELISA assay. Cells were washed with PBS and then collected at room temperature. Subsequently, a luciferase-based ATP assay kit (Celltiter-Glo Luminescent Cell Viability assay; Promega, Madison, WI, USA; Catalogue No. A22066) was used according to the instructions [39].

### Flow cytometry for mitochondrial ROS

Cell suspensions were collected. The liquor (50 g, digested two times) was collected, centrifuged for 2 min with the supernatant removed, supplemented with the MitoSOX red mitochondrial superoxide indicator (Molecular Probes, USA) [40], incubated at room temperature for 10 min, centrifuged, and washed with PBS. The cells were resuspended by adding binding buffer (1×) in the dark [41]; then, the cells were incubated at room temperature for 30 min and filtered with a nylon mesh (40 µm well). The ROS production was measured by fluorescence-activated cell sorting (FACS) [42].

### Statistical analysis

SPSS 21.0 software (IBM Corp., Armonk, New York, USA) was applied for data analysis. All experiments were repeated 3 times in each group. The mean value of the measurement data was expressed as the mean and SEM. Comparisons among groups were by one-way analysis of variance (ANOVA), and multiple comparisons between the average number of samples were performed by LSD analysis according to several previous studies [43, 44]. p < 0.05 indicated that the difference was statistically significant.

## Results

### LATS2 is downregulated after exposure to 5-FU and LATS2 overexpression enhances 5-FU-mediated apoptosis in SW480 cells

To examine the function of LATS2 in 5-FU resistance, western blotting was performed to observe changes in LATS2 in response to 5-FU treatment. As shown in Fig. 1a, b, compared to the control group, LATS2 was significantly downregulated in SW480 cells after exposure to 5-FU. This finding was also validated by qPCR. As shown in Fig. 1c, compared with the control group, 5-FU treatment markedly reduced the transcription of LATS2 in SW480 cells. Besides, cell viability was measured via MTT assay. As shown in Fig. 1d, compared to the control group, SW480 cell viability was reduced after exposure to 5-FU treatment. Because minimal 5-FU toxicity was observed at a concentration of 2 μg/ml, this concentration was used in the following studies. To further examine the effect of LATS2 loss in SW480 cells, adenovirus-loaded LATS2 was transfected into SW480 cells to reverse LATS2 expression in the presence of 5-FU treatment. The overexpression efficiency was confirmed via western blotting. As shown in Fig. 1e, f, compared to the 5-FU group, Ad-LATS2 transfection significantly reversed LATS2 expression in SW480 cells. Subsequently, cell viability was measured via an LDH release assay. As shown in Fig. 1g, compared to the control group, the content of LDH in the medium was rapidly increased in response to 5-FU treatment, indicating induction of cell membrane breakage by 5-FU. Interestingly, this alteration was enhanced by LATS2 overexpression.

The article "Large tumor suppressor kinase 2 overexpression attenuates 5-FU-resistance in colorectal cancer via activating the JNK-MIEF1-mitochondrial division pathway" was retracted in 2023. Reasons: duplicated images; signs of a paper mill; unreliable data; unreliable results or conclusions.

**Fig. 1:** 5-FU treatment attenuates the levels of LATS2 and overexpression of LATS2 enhances 5-FU-mediated cancer cell death in vitro. **a**–**b** Different doses of 5-FU were added into the medium of SW480 cells and then proteins were isolated from cells. Western blotting was used to observe the alterations of LATS2 in response to 5-FU treatment. **c** RNA was isolated from SW480 cells and then the transcription of LATS2 mRNA was evaluated via qPCR. 5-FU treatment dose-dependently reduced the transcription of LATS2 in SW480 cells. **d** Cellular viability of SW480 cells was determined via MTT assay. **e**, **f** LATS2 adenovirus vectors (ad-LATS2) were transfected into SW480 cells and then the overexpression efficiency of LATS2 was confirmed via western blotting. **g** After LATS2 was overexpressed, the cell death was evaluated via LDH release assay. LATS2 overexpression could further elevate the LDH content in the medium. **h** Caspase-3 activity was evaluated via ELISA. LATS2 adenovirus vectors (ad-LATS2) were transfected into SW480 cells. **i**, **j** TUNEL staining was used to label the apoptotic cells. The number of TUNEL-positive cell was recorded to reflect the cell death in response to LATS2 overexpression. *p < 0.05 vs. control (ctrl) group; #p < 0.05 vs. 5-FU + ad-ctrl group; ad-ctrl: control null adenovirus vectors; ad-LATS2: LATS2 adenovirus vectors

To further examine whether this cell death resulted from increased apoptosis, ELISA was used to analyse caspase-3 activity. Compared to the control group, the activity of caspase-3 increased rapidly in response to 5-FU treatment, and this effect was further enhanced by overexpression of LATS2 (Fig. 1h). This finding was further supported by TUNEL staining. As shown in Fig. 1i, j, compared to the control group, 5-FU treatment increased the ratio of TUNEL-positive cells. Interestingly, overexpression of LATS2 in the presence of 5-FU further elevated the number of TUNEL-positive cells, indicating that 5-FU-mediated cell apoptosis could be augmented via upregulation of LATS2 (Fig. 1i, j). Taken together, the above data indicated that the anti-apoptotic effect of 5-FU could be enhanced by LATS2 overexpression in SW480 cells.

The article "Large tumor suppressor kinase 2 overexpression attenuates 5-FU-resistance in colorectal cancer via activating the JNK-MIEF1-mitochondrial division pathway" was retracted in 2023. Reasons: duplicated images; signs of a paper mill; unreliable data; unreliable results or conclusions.

### SW480 cell proliferation and movement are affected by 5-FU and LATS2

To verify the role of LATS2 in cell proliferation and mobilization, EdU staining and Transwell assays were performed. As shown in Fig. 2a, b, EdU staining demonstrated that the number of EdU-positive cells was rapidly repressed in response to 5-FU treatment. Interestingly, 5-FU-mediated cell proliferation arrest was further enhanced by LATS2 overexpression, as evidenced by the deceased ratio of EdU-positive cells in SW480 cells (Fig. 2a, b). At the molecular level, cell proliferation is modulated by cyclin proteins such as CDK4 and Cyclin D1. As shown in Fig. 2c, e, compared to the control group, 5-FU treatment inhibited the expression of Cyclin D1 and CDK4. Interestingly, the combination of LATS2 overexpression and 5-FU treatment further repressed the levels of CDK4 and Cyclin D1 in SW480 cells (Fig. 2c, e). Therefore, the above data indicate that cyclin proteins are modulated by 5-FU and this effect is further enhanced by LATS2 overexpression.

**Fig. 2:** LATS2 overexpression augments 5-FU-mediated cell proliferation arrest and mobilization inhibition. **a**, **b** EdU staining was used to evaluate cell proliferation. The number of EdU positive cell was recorded. **c**–**e** Proteins were isolated from SW480 cells and then western blotting was used to evaluate the expression of cyclin D1 and CDK4. **f**, **g** Transwell assay was used to observe the number of migrated cells. **h**, **i** RNA was isolated from SW480 cells and then the expression of metastatic genes were evaluated via qPCR. *p < 0.05 vs. control (ctrl) group; #p < 0.05 vs. 5-FU + ad-ctrl group; ad-ctrl: control null adenovirus vectors; ad-LATS2: LATS2 adenovirus vectors

In addition to cell proliferation, Transwell assays demonstrated that the number of migrating cells decreased rapidly in response to 5-FU treatment (Fig. 2f, g). However, combining LATS2 overexpression with 5-FU treatment further inhibited the number of migrating cells (Fig. 2f, g). Subsequently, qPCR was used to observe alterations of metastatic genes such as ROCK1 and Rac. As shown in Fig. 2h, i, compared to the control group, ROCK1 and Rac transcription were significantly inhibited by 5-FU treatment, and this effect was enhanced by ad-LATS2 transfection. These results indicated that cellular movement is highly regulated by 5-FU in a LATS2-dependent manner.

The article "Large tumor suppressor kinase 2 overexpression attenuates 5-FU-resistance in colorectal cancer via activating the JNK-MIEF1-mitochondrial division pathway" was retracted in 2023. Reasons: duplicated images; signs of a paper mill; unreliable data; unreliable results or conclusions.

### Mitochondrial dysfunction is modulated by 5-FU and LATS2 in SW480 cells

Next, experiments were performed to analyse mitochondrial function in response to 5-FU treatment and LATS2 overexpression in SW480 cells. As shown in Fig. 3a, b, mitochondrial membrane potential, as assessed via the JC-1 probe, was rapidly downregulated in response to 5-FU treatment and LATS2 overexpression. Interestingly, the combination of 5-FU treatment and LATS2 overexpression further inhibited mitochondrial membrane potential (Fig. 3a, b), as evidenced by decreased red-to-green fluorescence intensity ratio. At the molecular level, the mitochondrial potential plays a decisive role in ATP production in cancer cells [44, 45]. Accordingly, ATP production was measured in SW480 cells. As shown in Fig. 3c, compared to the control group, 5-FU treatment repressed ATP content in SW480 cells, and this effect was further enhanced by LATS2 overexpression. Notably, the mitochondrial respiratory complex also participates in energy metabolism [46, 47]. Western blotting revealed that the expression of the mitochondrial respiratory complex was rapidly downregulated in response to 5-FU treatment, and this effect was further augmented by LATS2 overexpression (Fig. 3d–g). Taken together, the above data indicate that LATS2 overexpression aggravates 5-FU-mediated mitochondrial dysfunction in SW480 cells.

**Fig. 3:** Mitochondrial dysfunction is triggered by 5-FU treatment and this effect is further augmented by LATS2 overexpression. **a**, **b** Mitochondrial membrane potential was determined via JC-1 probe. Red fluorescence means the normal mitochondrial membrane potential whereas green fluorescence indicates the damaged mitochondrial potential. The red-to-green fluorescence ratio was used to quantify mitochondrial membrane potential. **c** Cellular ATP production was determined. LATS2 adenovirus vectors (ad-LATS2) were transfected into SW480 cells. **d**–**g** Proteins were isolated from SW480 cells and then the expression of mitochondrial respiratory complex was determined via western blotting. *p < 0.05 vs. control (ctrl) group; #p < 0.05 vs. 5-FU + ad-ctrl group; ad-ctrl: control null adenovirus vectors; ad-LATS2: LATS2 adenovirus vectors

The article "Large tumor suppressor kinase 2 overexpression attenuates 5-FU-resistance in colorectal cancer via activating the JNK-MIEF1-mitochondrial division pathway" was retracted in 2023. Reasons: duplicated images; signs of a paper mill; unreliable data; unreliable results or conclusions.

### LATS2 overexpression augments 5-FU-mediated mitochondrial apoptosis in SW480 cells

Excessive mitochondrial malfunction is associated with the initiation of mitochondrial apoptosis [7, 48, 49]. There are three molecular events in mitochondrial apoptosis: mitochondrial ROS accumulation, cyt-c release into the nucleus, and upregulation of mitochondrial apoptosis proteins [50–52]. Flow cytometry analysis revealed that the production of mitochondrial ROS was significantly increased in response to 5-FU treatment (Fig. 4a, b). However, the pro-oxidant effects of 5-FU were further enhanced by LATS2 overexpression (Fig. 4a, b). In addition to ROS overproduction, cyt-c translocation into the nucleus was evaluated by immunofluorescence assays. As shown in Fig. 4c, d, compared to the control group, a portion of cyt-c was translocated into the nucleus in response to 5-FU treatment. Interestingly, LATS2 overexpression facilitated 5-FU-mediated cyt-c translocation (Fig. 4c, d), as evidenced by the increase in nuclear cyt-c expression upon 5-FU treatment combined with LATS2 overexpression. Finally, western blotting was used to observe the alterations of mitochondrial apoptosis-related proteins. As shown in Fig. 4e–i, compared to the control group, 5-FU treatment elevated the expression of mitochondrial apoptosis-related proteins, as evidenced by increased caspse-9 and Bax. Interestingly, the levels of Bcl-2 and survivin were rapidly downregulated after exposure to 5-FU. Notably, LATS2 overexpression enhanced the upregulation of mitochondrial pro-apoptotic proteins mediated by 5-FU (Fig. 4e–i). Therefore, the above data indicate that 5-FU treatment induces mitochondrial apoptosis and that this effect is further amplified by LATS2 overexpression.

**Fig. 4:** 5-FU-activated mitochondrial apoptosis could be enhanced by LATS2 overexpression. **a**, **b** The levels of ROS were evaluated via flow cytometry. **c**, **d** Immunofluorescence assay for cyt-c translocation. The expression of nuclear cyt-c was determined to quantify mitochondrial apoptosis. **e**–**i** Proteins were isolated from SW480 cells and then the expression of mitochondrial apoptotic factors was evaluated via western blotting. *p < 0.05 vs. control (ctrl) group; #p < 0.05 vs. 5-FU + ad-ctrl group; ad-ctrl: control null adenovirus vectors; ad-LATS2: LATS2 adenovirus vectors

### MEF1-related mitochondrial division is further activated by LATS2 overexpression in the presence of 5-FU

Recent studies have shown that mitochondrial division is closely associated with cancer therapeutic response by increasing mitochondrial oxidative stress and activating caspase-9-related apoptotic pathways. MIEF1 is recently identified as a novel mediator of mitochondrial division. In the present study, we ask whether LATS2 overexpression enhances 5-FU-mediated SW480 cell damage by modifying MIEF1-related mitochondrial division. First, western blotting was performed to analyse the expression of mitochondrial division-related proteins. Drp1 and Mff are pro-division factors, whereas Mfn2 and Opa1 are anti-division proteins. As shown in Fig. 5a–f, compared to the control group, 5-FU treatment elevated the expression of Drp1 and Mff, an effect that was accompanied by an increase in MIEF1. By contrast, the levels of Mfn2 and Opa1 were rapidly downregulated in response to 5-FU treatment (Fig. 5a–f). Interestingly, the 5-FU-mediated imbalance between pro-division proteins and anti-division factors was further amplified by LATS2 overexpression (Fig. 5a–f). These results indicate that mitochondrial fission is initiated by 5-FU and that this effect is further enhanced by LATS2 overexpression.

The article "Large tumor suppressor kinase 2 overexpression attenuates 5-FU-resistance in colorectal cancer via activating the JNK-MIEF1-mitochondrial division pathway" was retracted in 2023. Reasons: duplicated images; signs of a paper mill; unreliable data; unreliable results or conclusions.

**Fig. 5:** Mitochondrial fission is modulated by 5-FU in a manner dependent on LATS2. **a**–**f** SW480 cells were treated with 5-FU and/or LATS2 overexpression. Then, proteins were isolated from cells and the expression of mitochondrial fission-related factors were evaluated via western blotting. LATS2 overexpression further upregulated 5-FU-activated mitochondrial fission factors. **g**, **h** Immunofluorescence assay for mitochondria. Mitochondrial morphology was observed, and then mitochondrial length was determined to quantify mitochondrial fission. *p < 0.05 vs. control (ctrl) group; #p < 0.05 vs. 5-FU + ad-ctrl group; ad-ctrl: control null adenovirus vectors; ad-LATS2: LATS2 adenovirus vectors

Subsequently, immunofluorescence assays were used to observe mitochondrial division based on a previous study [53, 54]. As shown in Fig. 5g, h, mitochondria in normal SW480 cells were rod-like, whereas 5-FU treatment caused mitochondrial fragmentation. Interestingly, this alteration was further enhanced by LATS2 overexpression. Then, mitochondrial length was measured as an indicator of mitochondrial division. As shown in Fig. 5g, h, the mitochondrial length decreased from ~ 9.5 μm to ~ 4.5 μm in response to 5-FU treatment. Interestingly, the combination of LATS2 overexpression with 5-FU treatment further reduced the mitochondrial length to ~ 3.3 μm (Fig. 5g, h). The above data indicate that MIEF1-related mitochondrial division is activated by 5-FU and that this effect is augmented by overexpression of LATS2.

The article "Large tumor suppressor kinase 2 overexpression attenuates 5-FU-resistance in colorectal cancer via activating the JNK-MIEF1-mitochondrial division pathway" was retracted in 2023. Reasons: duplicated images; signs of a paper mill; unreliable data; unreliable results or conclusions.

### MIEF1-related mitochondrial division is required for 5-FU/LATS2-mediated mitochondrial damage and cell death

To determine if MIEF1-related mitochondrial division is responsible for 5-FU/LATS2-mediated mitochondrial damage and cell death, siRNA against MIEF1 was transfected into 5-FU/LATS2-treated cells (Fig. 6a, b) [55]. The knockdown efficiency was confirmed via western blotting (Fig. 6a, b). Then, mitochondrial function was determined via immunofluorescence [56]. As shown in Fig. 6c, d, compared to the control group, 5-FU in combination with LATS2 overexpression promoted cyt-c translocation into the nucleus, and this effect was reversed by MIEF1 knockdown. In addition to cyt-c translocation, ELISA was performed to observe alterations of cellular antioxidants. As shown in Fig. 6e–g, compared to the control group, the levels of SOD, GSH and GPX were rapidly downregulated in response to 5-FU and LATS2 overexpression. Interestingly, loss of MIEF1 could reverse the levels of cellular antioxidants. Finally, caspase-9 activity was measured as an indicator of mitochondrial damage. As shown in Fig. 6h, compared to the control group, the activity of caspase-9 was significantly elevated in response to 5-FU/LATS2 overexpression, and this effect was negated by MIEF1 knockdown. Therefore, the above data indicate that MIEF1 is required for 5-FU/LATS2-mediated mitochondrial stress.

**Fig. 6:** LATS2 overexpression affects 5-FU-triggered mitochondrial fission via MIEF1. **a**, **b** Proteins were isolated from SW480 cells and then the expression of MIEF1 was determined via western blotting. siRNA against MIEF1 was transfected into 5-FU/LATS2-treated SW480 cells. **c**, **d** Immunofluorescence assay for cyt-c. The expression of nuclear cyt-c was determined. **e**–**g** Cellular anti-oxidants were determined via ELISA. siRNA against MIEF1 was transfected into 5-FU/LATS2-treated SW480 cells. **h** Caspase-9 activity was evaluated via ELISA. siRNA against MIEF1 was transfected into 5-FU/LATS2-treated SW480 cells. **i** The content of LDH in the medium was evaluated via ELISA. SW480 cells were treated with 5-FU and/or transfected with LATS2 adenovirus. siRNA against MIEF1 was transfected into 5-FU/LATS2-treated SW480 cells. *p < 0.05 vs. control (ctrl) group; #p < 0.05 vs. 5-FU + ad-ctrl group; @p < 0.05 vs.5-FU + ad-LATS2 + si-ctrl group; ad-ctrl: control null adenovirus vectors; ad-LATS2: LATS2 adenovirus vectors; si-MIEF1: siRNA against MIEF1

The role of MIEF1-related mitochondrial division in cell death was analysed by performing LDH release assays [57]. As shown in Fig. 6i, compared to the control group, the content of LDH in the medium was rapidly increased in response to 5-FU/LATS2 overexpression, and this effect was abolished by MIEF1 siRNA. Taken together, our results confirm the essential role of MEIF1-related mitochondrial division in 5-FU/LATS2 overexpression-mediated mitochondrial malfunction and cell death.

The article "Large tumor suppressor kinase 2 overexpression attenuates 5-FU-resistance in colorectal cancer via activating the JNK-MIEF1-mitochondrial division pathway" was retracted in 2023. Reasons: duplicated images; signs of a paper mill; unreliable data; unreliable results or conclusions.

### 5-FU/LATS2 modulates MIEF1 via the JNK pathway

We next sought to determine the molecular mechanism by which 5-FU/LAT2 affects MIEF1-related mitochondrial division in SW480 cells. Previous studies have found that the JNK pathway is an upstream mediator of mitochondrial division by controlling mitochondrial division-related proteins such as Drp1, Mff and Opa1 [58, 59]. Accordingly, we examined whether the JNK pathway was also involved in MIEF1 expression induced by 5-FU/LATS2 overexpression. As shown in Fig. 7a–c, compared to the control group, the expression of p-JNK was markedly increased in response to 5-FU/LATS2 overexpression, an effect that was accompanied by an augmentation of MIEF1 expression. Interestingly, inhibition of the JNK pathway using SP600125 significantly repressed p-JNK expression concomitant with a decrease in MIEF1 expression in the presence of 5-FU treatment and LATS2 overexpression. These results indicated that the JNK pathway, activated by 5-FU/LATS2 overexpression, was required for the upregulation of MIEF1 in SW480 cells. This finding was further supported by the results of immunofluorescence assays. As shown in Fig. 7d–f, compared to the control group, the fluorescence intensity of p-JNK and MIEF1 were rapidly elevated in response to 5-FU/LATS2 overexpression; this effect was largely abrogated by SP600125, a specific inhibitor of the JNK pathway. Taken together, the above data indicate that MIEF1 is modulated by 5-FU/LATS2 overexpression via the JNK pathway.

**Fig. 7:** 5-FU/LATS2 controls MIEF1 expression via the JNK pathway. **a**–**c** SW480 cells were treated with 5-FU and/or transfected with LATS2 adenovirus. SP600125 was used to inhibit the JNK activation. Proteins were isolated from SW480 cells and then the expression of p-JNK and MIEF1 was determined via western blotting. **d**–**f** Immunofluorescence assay for p-JNK and MIEF1. The fluorescence intensity of p-JNK and MIEF1 was determined. SP600125 was used to inhibit the JNK activation. *p < 0.05 vs. control (ctrl) group; #p < 0.05 vs. 5-FU + ad-ctrl group; @p < 0.05 vs.5-FU + ad-LATS2; ad-ctrl: control null adenovirus vectors; ad-LATS2: LATS2 adenovirus vectors

## Discussion

Colorectal cancer (CRC), one of the most common malignancies, account for 48% of colon-related deaths. 5-FU treatment is the standard approach to control the progression of CRC, but acquired resistance and/or a low therapeutic response remain major challenges in clinical practice. More than half of CRC patients develop therapeutic resistance through mechanisms that are poorly understood. Accordingly, there is an urgent need to elucidate the molecular mechanism underlying drug resistance. In the present study, we found that LATS2, a component of the Hippo pathway, was significantly repressed by 5-FU treatment. Interestingly, overexpression of LATS2 further enhanced 5-FU-mediated SW480 cell death in vitro. Molecular investigations demonstrated that 5-FU treatment was associated with cell apoptosis, proliferation arrest, movement inhibition, and mitochondrial dysfunction. Interestingly, overexpression of LATS2 elevated 5-FU-mediated mitochondrial division in a manner dependent on MIEF1. Excessive MIEF1-related mitochondrial division exacerbated mitochondrial damage and amplified 5-FU-induced apoptosis in SW480 cells. However, loss of MIEF1 via transfection of siRNA abolished the pro-apoptotic effects of 5-FU and LATS2 overexpression. Accordingly, our results highlight that 5-FU resistance in SW480 cells is associated with LATS2 downregulation. This investigation is the first to explore the relationship between 5-FU resistance and the LATS2-Hippo pathway with a focus on MIEF1-related mitochondrial division. The findings of this study will pave the way for new strategies to augment 5-FU-based therapy in patients with CRC.

The article "Large tumor suppressor kinase 2 overexpression attenuates 5-FU-resistance in colorectal cancer via activating the JNK-MIEF1-mitochondrial division pathway" was retracted in 2023. Reasons: duplicated images; signs of a paper mill; unreliable data; unreliable results or conclusions.

A number of studies have shown that activation of mitochondrial division greatly elevates the cancer cell death ratio and inhibits tumour metastasis. Cancer metabolism preference, cyclin-mediated cell proliferation, mitophagy flux, mitochondrial bioenergetics, and chemotherapy resistance are also regulated by mitochondrial division [60]. At the molecular level, mitochondrial division produces massive amounts of mitochondrial fragments containing damaged DNA and reduces the mitochondrial membrane potential [61, 62]. These mitochondrial fragments contribute to an overload of reactive oxygen species (ROS), which mediates cancer oxidative stress [59, 63]. Mitochondrial division also promotes the opening of mitochondrial permeability transition pore (mPTP), a hallmark of mitochondrial death [64]. In addition, fragmented mitochondria cannot produce enough ATP for cancer metabolism. According to the above mechanisms, mitochondrial division has been identified as a potential target for further augmenting cancer death. In the present study, mitochondrial division was elevated by 5-FU, and overexpression of LATS2 furtherer amplified this increase in mitochondrial division in an MIEF1-dependent manner. This result indicates that the therapeutic sensitivity of 5-FU is modulated by LATS2 via MIEF1-related mitochondrial division. Besides, our data provide new insights for overcoming 5-FU resistance by targeting MIEF1-related mitochondrial division and LATS2. This finding might be helpful for the drug development for the CRC patients.

The article "Large tumor suppressor kinase 2 overexpression attenuates 5-FU-resistance in colorectal cancer via activating the JNK-MIEF1-mitochondrial division pathway" was retracted in 2023. Reasons: duplicated images; signs of a paper mill; unreliable data; unreliable results or conclusions.

MIEF1 is a novel mitochondrial division mediator. In Alzheimer’s disease [65], cardiac ischemia reperfusion injury, and ultraviolet irradiation-induced epidermal injury [9], MIEF1-related mitochondrial division is closely associated with cell viability and mitochondrial apoptosis. At the molecular level, MIEF1 helps Drp1 translocate from the cytoplasm into the surface of mitochondria. Subsequently, with the aid of MIEF1, Drp1 forms the contractile ring around mitochondria that ultimately mediates mitochondrial division. Endoplasmic reticulum (ER) stress and mitochondrial biosynthesis [66] also appear to be modulated by MIEF1. In the present study, we identified MIEF1 as a downstream effector of 5-FU and LATS2. An increase in MIEF1 is required for 5-FU-mediated mitochondrial malfunction and SW480 cell death. This result identifies 5-FU/LATS2/MIEF1 as a new signalling pathway regulating CRC viability by affecting mitochondrial division.

Furthermore, we determined that the JNK pathway is employed by LATS2 and/or 5-FU to modulate MIEF1-related mitochondrial division. The anti-cancer effects of JNK have been widely explored. The JNK pathway is a classic pathway responsible for the modification of mitochondrial division. In the present study, we found that JNK inhibition largely abolished the cancer-killing effects of 5-FU and LATS2 overexpression, supporting the functional importance of JNK as a key mediator transmitting damage signals from 5-FU into mitochondria with the help of mitochondrial division.

## Conclusions

In summary, our studies reveal that LATS2 overexpression can enhance the therapeutic efficiency of 5-FU by augmenting mitochondrial stress in a manner dependent on mitochondrial division. Mechanistically, LATS2 overexpression helps 5-FU further activate the JNK pathway, which increases the expression of MIEF1, thereby amplifying fatal mitochondrial division. This finding provides evidence that LATS2 overexpression could overcome 5-FU resistance by augmenting MIEF1-related mitochondrial division via JNK.

## Abbreviations

mROS: mitochondrial reactive oxygen species
LATS2: large tumor suppressor kinase 2
mPTP: mitochondrial permeability transition pore
MIEF1: mitochondrial elongation factor 1
